# Improving boron use efficiency via different application techniques for optimum production of good quality potato *(Solanum tuberosum* L.) in alkaline soil

This article has been retracted.

**DOI:** 10.1371/journal.pone.0259403

**Published:** 2022-01-27

**Authors:** Muhammad Tariq, Bilal Ahmad, Muhammad Adnan, Ishaq Ahmad Mian, Shadman Khan, Shah Fahad, Muhammad Hamzah Saleem, Mukhtiar Ali, Maria Mussarat, Manzoor Ahmad, Muhammad Romman, Muhammad Sohaib Chattha, Mohamed A. El-Sheikh, Shafaqat Ali

**Affiliations:** 1 Department of Soil and Environmental Sciences, University of Agriculture, Peshawar, Khyber Pakhtunkhwa, Pakistan; 2 Department of Agriculture, University of Swabi, Swabi, Khyber Pakhtunkhwa, Pakistan; 3 Department of Agronomy, University of Haripur, Haripur, Khyber Pakhtunkhwa, Pakistan; 4 College of Plant Science and Technology, Huazhong Agricultural University, Wuhan, China; 5 Department of Soil Science, Nuclear Institute for Food and Agriculture (NIFA), Peshawar, Khyber Pakhtunkhwa, Pakistan; 6 Department of Agriculture, Bacha Khan University, Charsadda, Khyber Pakhtunkhwa, Pakistan; 7 Department of Botany, University of Chitral, Chitral, Khyber Pakhtunkhwa, Pakistan; 8 School of Plant, Environmental, and Soil Sciences, Louisiana State University Agricultural Center, Baton Rouge, LA, United States of America; 9 Botany & Microbiology Department, College of Science, King Saud University, Riyadh, Saudi Arabia; 10 Department of Environmental Sciences and Engineering, Government College University, Faisalabad, Punjab, Pakistan; 11 Department of Biological Sciences and Technology, China Medical University (CMU), Taichung City, Taiwan; Anhui Agricultural University, CHINA

## Abstract

Boron (B) deficiency is a widespread problem in alkaline soils which affects yield and quality of potato but is often ignored by the growers. That’s why, we compared the impact of different methods of boron application (foliar spray, fertigation and soil dressing) along with control on boron use efficiency (BUE), quality and yield of potato in alkaline soils. Boron (0.5 kg ha^-1^) applied as a foliar spray had significantly increased plant height, tuber per plant, tuber volume and enhanced the quality in terms of vitamin C, starch and B content of potato compared to other methods. Moreover, foliar applied B significantly improved B uptake and it use efficiency over other application methods. B concentration in tubers were strongly correlated with vitamin C and starch contents. The application methods were ranked as foliar spray>fertigation>soil dressing in term of their effectiveness towards potato yield and quality improvement. Thus, for optimum production of good quality potato, B should be applied as foliar spray at the rate of 0.5 kg B ha^-1^ in existing agro-climatic conditions.

## 1. Introduction

Potato (*Solanum tuberosum* L.) is an important cash crop in the world and is used in many commercial food products such as French fries, chips and starches [1]. it is a good source of carbohydrates, and vitamins [2]. Potato growth and productivity can be severely influenced by abiotic stresses like nutrients and water deficiency, high temperature, strong wind and exposure to UV(ultra violet) radiation. The judicious use of fertilizers and proper placement method is the best approach for enhancing potato productivity [3].

Boron (B) is a micro essential plant nutrient and is deficient in light and alkaline soils, having low organic matter and high pH [4, 5]. Its deficiency is a main yield limiting factor in potato productivity in Pakistan. Beneficial effects of B application to soil have been reported by several researchers. Shirur et al. [6] obtained maximum fresh weight, tuber number, dry matter content and potato tuber yield with incorporation of 1.1 kg B ha^-1^ in alkaline soil. Boron is slowly released from soil because it is tied up by soil organic matter and only becomes available with the decomposition [7].

Foliar application of B is an effective approach for fulfilling boron requirement due to better absorption through leaves [8, 9]. Nutrients are more available to the plants by the foliar spray than conventional fertilization application [10]. Nutrients apply as foliar gives 90% more efficient results as compare to surface application [11, 12]. According to Khan et al. [13], in sandy loam soil, foliar application is up to 20% more efficient in comparison to soil applied fertilizer. Similarly, Supplying B in the irrigation water is advantageous over broadcast application to soil [14]. Furthermore, foliar application ensures timely nutirent availability, reduce losses and prevent environmental contimination [15].

Mismanagement of nutrients can lead to soil and water contamination and degraded soil [16]. However, fertigation serve best in this regard by improving nutrient use efficiency and ensure more availability of nutrients [17]. Boron is a mobile nutrient in soil system that is why, it reaches roots by mass flow, while its translocation in plants is governed by the transpiration stream through the xylem [18]. In plants boron is immobile, and thus its accessibility is indispensable at all growth stages, especially during fruit/seed development stage.

Much more work has done on exploring the role of B on potato yield and quality but little is known regarding its application methods and their impact on quality and B use efficiency. We assumed that foliar B application is the best option for improving B availability in alkaline calcareous soils. Therefore, this study was carried out to compare the efficacy of different boron application methods like foliar, soil application and fertigation for improving yield, quality and B use efficiency of potato crop.

## 2. Materials and methods

### 2.1. Experimental location

The field study was carried out at Nuclear Institute of Food and Agriculture (NIFA), Peshawar-Pakistan in spring 2018. The soil of experimental site was silt loam in texture, alkaline. non saline and calcareous in nature, low in organic matter and plant available boron as shown in Table 1. The field study was carried out at Nuclear Institute of Food and Agriculture (NIFA), Peshawar-Pakistan in spring 2018 (34° 0’56.35"N 71°42’45.86"E). The Director NIFA (Dr. Wisal Muhammad) allowed us to use their field and laboratory on the request of the chairman Department of Soil and Environmental Sciences, The University of Agriculture Peshawar.

**Table 1:** Physico-chemical properties of the experimental soil.

Property	Unit	Value
Soil Texture	-	Silt loam
pH _**(1:5)**_	-	8.25
E.C _**(1:5)**_	dSm^-1^	0.62
CaCO_3_	%	13.3
Organic matter	%	1.05
HWS-boron	mg kg^-1^	0.24

### 2.2. Experimental layout and sowing

This field study was carried out in randomized complete block design with three replication. The experiment was comprised of different methods of boron application such as soil dressing, foliar application, fertigation along with control. Potato variety *Racco* was sown on 18^th.^ February, 2018. Boron was applied at the rate of 1 kg ha^-1^ as side dressing and fertigation, whereas foliar boron was applied in 0.5 kg B ha^-1^. For soil dressing, borax was mixed with the soil and applied as side dressing to the respective treatment plots after the sowing of seed potato. For foliar spray, the spray solution was prepared from commercial borax fertilizer available in the market. Fertigation was done by calculating amount of borax and was dissolved in water and applied with irrigation water. Boron fertigation was done two times with irrigation. Boron application as foliar spray was applied two times during experiment, one at vegetative stage and the other at tuber formation stage of the crop.

Recommended dose of nitrogen, phosphorus and potassium (NPK) was applied to each treatment plot at the ratio of 220:120:60 kg ha^-1^. Before the preparation of seedbed all the P and K were amended from di-ammonium phosphate, potassium sulphate, respectively, while N was applied as urea in two (2) split doses, one at sowing time and second at flowering stage of the crop was given. Size of the plot was kept 15 m^2^ consisting of 6 rows in every treatment, while the space between rows was maintained 80 cm. All other agronomic practices like irrigation, weeding was practiced uniformly in each treatment plot during growth season.

### 2.3. Estimation of yield and yield traits

Plant height was recorded 70 days after the sowing by randomly selecting 5 plants from every treatment plot and was measured from the tip of the plant to its base. The gross yields of haulm plot^-1^ were recorded after harvesting and were expressed in kilogram. Finally, the yield was converted to t ha^-1^ on dry basis. At harvesting stage, number of tuber plant^-1^ were recorded by counting the tuber number of 5 randomly selected plants in each treatment plot for each replication and their average was calculated. The volume of three randomly selected potatoes was measured by the help of water displacement method [18]. The change in volume was considered as the volume of selected potato as calculated by the Eq 1, as below:

$$Volume\;({cm}^{3})=\frac{\left(final\;volume–initial\;volume\right)}{Number\;of\;potato}\times \frac{{cm}^{3}}{mL}$$ (1)

### 2.4. Quality attributes

Vitamin C (mg/100g) in the samples was processed by the AOAC method [19]. The determination of the starch content of the sample was measured by the method of Zeng et al. [20]. Boron concentration in plants was measured by collected at flowering stage of crop. The leaves, stem and tuber were washed with distilled water and were ashed in furnace at 550 C0 then dissolved in 0.5 M HCl and passed through filter paper [21]. The collected sample was subjected to Azomethine-H color development Hendrey [22] by using spectro-photometer at 420 nm it reading was recorded. Boron uptake was quantified as the product of concentration and biomass of each treatment plot and was converted into kg ha^-1^. The moisture loss was found with the help of following Eq 2.


$$Moisture\;loss\;(\%)=\frac{initial\;wt-final\;wt}{initial\;wt}\times 100$$ (2)

The procedure of Crawswell [23] was used for the determination of B use efficiency by the following Eq 3.


$$Apparent\;nutrient\;recovery\;(\%)=\frac{{nutrient\;uptake}_{F}-{nutrient\;uptake}_{c}}{nutrient\;applied}\times 100$$ (3)

### 2.5. Statistical analysis

The collected data was analysed for analysis of variance (ANOVA) using Statistix 8.1 software. In addition, multiple regression analysis was performed between the yield, quality and boron concentration in various plant parts of potato crop [24].

## 3. Results

### 3.1. Potato yield and yield attributes

Boron application regardless of its application methods significantly affected the plant height, Biological yield, tubers per plant and tubers volume of potato (Table 2). Means table showed that plots treated with foliar application had resulted in taller plants followed by fertigation and then soil dressed boron. Whereas, the lower plant height was observed in control plot. Higher biological yield was obtained from those plots receiving B as foliar spray than fertigation followed by soil dressing, while lower was observed in control. Mean values indicated that foliar application gives higher number of tuber plant^-1^ followed by boron fertigation which was not statistically different from boron applied through soil application. The minimum number of tubers plant^-1^ was observed in control plots. Results regarding tuber size indicated that foliar application produced maximum size potato followed by boron applied through fertigation and soil application the latter two methods were at par while, the control plots produced smaller size of potato tuber.

**Table 2:** Effect of different application methods of boron on plant height (cm), number of tubers, biological yield (kg ha^-1^) and tuber volume of potato crop.

Application Methods	B (kg ha^-1^)	Mean			
		Plant height (cm)	Number of tuber (plant^-1^)	Biological yield (kg ha^-1^)	Tuber volume (cm^3^)
Control	0	48.92± 3.66b	5.00 ± 0.34 c	315.3 ± 36.96	81.11± 2.34 c
Foliar	0.5	56.67±5.47a	7.06 ± 0.64 a	391.0 ± 42.56	98.33± 1.67 a
Fertigation	1	55.08±2.88a	6.11 ±0.39 b	388.7 ± 15.53	90.22 ± 2.87 b
Soil	1	52.0±4.72ab	5.66 ± 0.34 bc	332.3 ± 22.48	88.88± 5.09 b
LSD (P<0.05)		9.62	1.17	109.35	10.86
CV (%)		5.74	5.67	8.85	3.50

Means followed by similar letter’s within the same category are statistically similar using LSD at P <0.05. The ± values represent standard error for mean (n = 3).

### 3.2. Quality attributes and boron use efficiency

Analysis of variance showed that boron application had significantly influenced the vitamin C, starch and moisture contents of potato tubers (Table 3). Maximum vitamin C content was obtained at foliar B spray which was statistically at par to fertigation. Whereas, the minimum vitamin C were observed from the control where no boron was applied and it was comparable to to plot receiving B as soil application. The maximum value of starch content in tubers was obtained in plots where B was suplimented as foliar application followed by fertigation and then soil application of boron. Whereas, the minimum starch content was observed in control. Means data showed that loss of weight in grams per week was maximum in control plot followed by boron applied through soil application which is statistically at par to one another (Fig 1). Loss in weight of the tuber in grams per week in fertigation and foliar application of boron are statistically same. However, loss of weight in fertigation of boron is slightly greater than boron applied through foliar application (Fig 1). Results show among the different methods of boron application, foliar spray gave maximum 25.62% boron recovery than boron applied through fertigation and soil dressing (Table 3).

**Fig 1:** Comparative effect of boron application methods on the boron use efficiency of potato crop.

**Table 3:** Effects of boron application methods on starch and vitamin C contents and boron use efficiency of potato crop.

Application methods	B (kg ha^-1^)		Mean		
			Starch (mg g^-1^)	Vitamin C (mg 100g^-1^)	Moisture loss (%)
Control		0	448.30±76.50 b	15.00 ± 0.29 c	34.40± 1.29a
Foliar		0.5	656.53±112.50a	17.50 ± 0.90 a	21.65±2.13 c
Fertigation		1	600.48± 85.80a	16.68 ±0.55 ab	25.18±1.26 c
Soil		1	570.27±3.16 a	15.92 ± 0.25 bc	29.88±2.87 b
LSD (P<0.05)			178.53	2.24	7.76
CV (%)			9.07	3.97	8.07

Means followed by similar letter’s within the same column are statistically similar using LSD at P <0.05. The ± values represent standard error (n = 3).

### 3.3. Boron concentration in leaves, stem and tubers and its uptake

Boron concentration in leaves, stem and tuber were significantly influenced by boron application methods (Table 4). Maximum boron concentration was observed in plots having foliar application of boron followed by boron applied through fertigation which are not statistically different with one another. Boron application increased the concentration of boron in stem as compared to control plot. However, there is no significant difference among foliar application and fertigation but foliar application was statistically different from soil applied boron. Foliar application resulted maximum boron concentration in stem followed by fertigation and then soil application while lower boron concentration was observed in control. Boron applied through foliar spray has significantly increased the boron concentration in tubers followed by fertigation as well as soil application. Analysis of the data clearly indicated that there was non-significant difference among boron applied through soil and fertigation, but boron fertigation gives slightly high value to that of soil application. Foliar application of boron resulted in maximum concentration, while lower concentration recorded in control plot.

**Table 4:** Effects boron application methods on boron concentration in leaves, stem, tuber and its uptake by potato crop.

Application methods	B (kg ha^-1^)	Mean			
		B conc. in leaves	B conc. in stem	B conc. in tuber	B uptake (g ha^-1^)
Control	0	46.67±10.00 b	45.00±3.51c	30.00 ±2.88c	103.03±14.03c
Foliar	0.5	75.00±21.79a	62.67±6.80a	46.67±5.77a	231.13±16.86a
Fertigation	1	65.00±8.66ab	55.56 ±6.03ab	38.33 ±7.64b	170.33±28.84b
Soil	1	55.00±5.03b	51.42± 2.64bc	36.67±5.00b	144.13±15.28b
LSD (P<0.05)		32.15	12.19	9.56	54.67
CV (%)		15.38	6.56	7.29	3.50

Means followed by similar letter’s within the same column are statistically similar using LSD at P <0.05. The ± values represent standard error (n = 3).

Simillarly, maximum B uptake was recorded for foliar spray, followed by fertigation and soil application (Table 4). Different methods of boron application linearly enhanced the total uptake of boron by plants with respect to control. The latter two methods were found statistically at par to one another while, minimumuptake was recorded in control plots.

### 3.4. Relationship between quality parameters and B concentration

Based on regression analysis vitamin C, moisture loss and starch content was correlated with boron concentration in tuber as presented in (Figs 2–4) respectively. These findings clearly indicated that as the boron concentration in tuber increased, the vitamin C is linearly increased and showed close relationship (r^2^ = 0.99) with each other. It was also evident that as the boron concentration in tuber increased, the loss of moisture in tuber linearly decreased and showed a close relationship (r^2^ = 0.99) with each other, indicating boron applied by various methods reduced the moisture losses of potato tuber as compared to control (where no boron was applied). Furthermore, the results indicated that as boron concentration in tuber increased, the starch content was also linearly increased and showed close relationship (r^2^ = 0.92) with each other.

**Fig 2:** Relationship of vitamin C (mg 100g^-1^) and B concentration in potato tuber.

**Fig 3:** Relationship between moisture loss and boron concentration in potato tuber.

**Fig 4:** Relationship of starch concentration (mg g^-1^) and B concentration in potato tuber.

## 4. Discussions

The height of the plant may be a genetic trait but proper nutrients, and soil and environmental condition also play a significant role in its enhancement. The plant height was significantly affected by boron application methods. Foliar spray of boron had resulted in taller plants than fertigation and soil applied boron. This increase in plant height might be due to the enlargement of cell wall which happen by the application of boron and it also help in the roots development of plants [25, 26] and increased the availability of NPK which improved the nutrition of potato plants and thus increased the plant height. These findings are in line with Jafari-Jood et al. [27], Rab and Haq [28], who stated that foliar application of boron improved plant height of potato plants. These results are in mutual agreement to the findings of [7, 27] who investigated that boron foliar spray in split doses to annual crops in term of vegetative growth were found superior to the soil dressing of boron.

Foliar application of boron was found superior in term of producing biological yield the treatments. This higher biological yield could be attributed to higher plant height which is an important contributing factor to biomass production [12, 29]. The present results suggested that the above ground portion of the potato crop was considerably increased due to foliar spray than other methods of boron placement [30]. As boron was effectively absorbed by leaves, and hence increased fresh biomass of potato crop [31]. These findings in contrast to recent work of [32], who urged that no significant differences were observed between soil and foliar applied boron on biological yield of potato tuber.

The yield of potato crop depends upon the number of tubers plant^-1^. Setting of tubers is greatly influenced by the rapid development and growth of leaves at flowering. Foliar spray of boron increased the number of tubers per plant this might be because of the greater accessibility of boron by foliar feeding and the important role of boron on sugar transport, increasing respiration rate and cell integrity, increasing uptake of some nutrients and metabolic activities [33]. Kaya et al. [34] found that foliar spray of boron increases the number of fruits in tomato. Our results agreed with recent work of Suganiya and Kumuthini [35] who observed maximum number of fruits plant^-1^ brinjal crop due to foliar application of 150 mg B L^-1^ than other treatment plots.

Foliar application of boron increased the size of potato tubers. This might be due to the fact that better mineral utilization of plants improved fruit weight and size by increasing photosynthetic efficiency. Bajapai and Chauhan [36] concluded that the weight and fruit size of okra (Abelmoschus esculentus) was increase by the foliar application of micronutrients. And Leghari et al. [37] also observed that split application of boron through foliar spray increased the seed size of mustard, wheat and potato crop.

Boron plays a significant role in the development of new cells, in meristem formation and plant growth, thus improve the fruit quality and fruit sets [31]. It also plays a greater role in the translocation of carbohydrates from leaves to other parts of the plants, greater ascorbic acid concentration may have been translocated to the tubers [38]. During the growth of potato plants, use of boron through foliar spray significantly increased the ascorbic acid concentration and made the tuber more nutritious and improved the overall tuber quality [1]. Besides the potato; boron also improved the quality of other crops like Hajduk et al. [30] reported maximum ascorbic acid (Vitamin C) content in tomato (32.57 mg/100g) with the foliar application of 1.25 g/L B.

Our findings of moisture loss are in accordance with Salam et al. [39] who reported that boron applied through foliar or through drip irrigation increase the shelf life of tomato crop which were statistically similar to each other. In foliar B application the loss in weight was low compared to control plot [8], suggested that the potato shelf life was increased due to foliar application of boron. The recent work of Shnain et al. [40] supported our findings, who observed that maximum shelf life of tomato fruit was due to foliar application of boron at the rate of 1.25 g L^-1^. The present results also suggest that boron applied through any method reduced the loss of water from potato tubers, because boron helps to maintain membrane stability [32] and perhaps boron also created firmness in the potato tubers [4, 6].

The increase in starch content of tubers might be attributed to the importance of micronutrients in carbohydrates metabolism, increasing the intensity of photosynthesis and the activity of oxidation-reduction enzymes [41]. These results are in line with the recent work of El-Dissoky [42] who reported that starch content increased by 25.83% with the application of boron. Foliar application of boron enhances quality of potato tuber like starch and vitamin C. Same results were also reported by El-Hoseiny [42] who noticed that starch content exerted significant influence to foliar application of humic acid, zinc and boron either alone or in combined treatment on pungent pepper.

The results of higher boron concentration in leaves is due to the fact that foliar applied boron efficiently enhanced boron concentration, while boron applied through soil mostly remained in the roots and a little of that was translocated to the upper parts of plants. These results are according with the findings of [3, 43] who documented that foliar application of boron enhances leaf boron content and improved transportation of boron to assorted growing parts. Furthermore, the latter authors observed that elevated boron concentration in leaves with foliar feeding over soil application. Boron concentration in stem was considerably influenced with application of boron. These results are in agreement with El-Dissoky [42] who noticed that foliar spray of boron increased the concentration of boron in stem of potato from 17.89 μg g^-1^. The results are also related to boron concentration are in accordance with Soomro, et al. [44] who found that maximum concentration of boron in maize straw at 0.5% foliar spray, applied at early, mid and late whorl stages an increase of 18.7% over control followed by soil application of boron.

Generally, application of boron through foliar spray have long been known to be an effective means of increasing boron concentration of the reproductive organs resulting in higher crop yield [45, 46]. These results are also in accordance with Sarkar, et al. [47], who observed that foliar spray of boron increased the boron concentration by 80% in potato tuber over the control plot. Boron use efficiency was considerably higher with foliar application than rest of the treatments. These findings suggest that foliar spray of boron is more effective in terms of maximum yield, good quality and nutrient uptake by potato crop under experimental condition. These results are in line with previous work of [46].The foliar application of B has long been known to be an effective means of enhancing the uptake of boron concentration in the aerial and reproductive organs producing higher crop yield [27] and immobility with in plants, once accumulated does not translocated [37]. These results are accordance with the previous work of Akter [48], who noticed that boron fertilization through foliar spray in potato increase overall boron uptake 10-fold or more than that by mustard or wheat because of its higher biomass yield. However, our findings are opposed to the recent work of Akter [48] who claimed that no significant effect of boron either soil or foliar application on the total uptake of boron by potato plants. The reason between the contradiction between the Akter [48] findings and present results mainly seems to be due to the application of boron along with zinc in Akhter’s experiment. Because zinc create protective mechanism against boron.

## 5. Conclusions

Potato yield and qualitative traits like vitamin C, starch content, boron concentration in leaves, stem, tuber and boron uptake were significantly improved with 0.5 kg B ha^-1^ applied as a foliar spray compared to other application methods. Vitamin C and strach contents were positvely correlated (r^2^ = 0.99 and 0.92 respectively) while, moisture loss was negetively correlated (r^2^ = 0.99) with boron concentration in tuber. Methods were ranked as, foliar spray > fertigation > soil dressing in terms of effectiveness. Therefore, boron should be applied at the rate of 0.5 kg ha^-1^ as foliar spray for optimum production of good quality potato in alakline soils.
